# iTAGPred: A Two-Level Prediction Model for Identification of Angiogenesis and Tumor Angiogenesis Biomarkers

**DOI:** 10.1155/2021/2803147

**Published:** 2021-09-27

**Authors:** Khalid Allehaibi, Yaser Daanial Khan, Sher Afzal Khan

**Affiliations:** ^1^Department of Computer Science, Faculty of Computing and Information Technology, King Abdulaziz University, Jeddah, Saudi Arabia; ^2^Department of Computer Science, University of Management and Technology, Lahore, Pakistan; ^3^Department of Computer Sciences, Abdul Wali Khan University Mardan, Pakistan

## Abstract

A crucial biological process called angiogenesis plays a vital role in migration, growth, and wound healing of endothelial cells and other processes that are controlled by chemical signals. Angiogenesis is the process that controls the growth of blood vessels within tissues while angiogenesis proteins play a significant role in the proper working of this process. The balancing of these signals is necessary for the proper working of angiogenesis. Unbalancing of these signals increases blood vessel formation, which causes abnormal growth or several diseases including cancer. The proposed work focuses on developing a two-layered prediction model using different classifiers like random forest (RF), neural network, and support vector machine. The first level performs in silico identification of angiogenesis proteins based on the primary structure. In the case the protein is an angiogenesis protein, then the second level predicts whether the protein is linked with tumor angiogenesis or not. The performance of the model is evaluated through various validation techniques. The model was evaluated using *k*-fold cross-validation, independent, self-consistency, and jackknife testing. The overall accuracy using an RF classifier for angiogenesis at the first level was 97.8% and for tumor angiogenesis at the second level was 99.5%, ANN showed 94.1% accuracy for angiogenesis and 79.9% for tumor angiogenesis, and the accuracy of SVM for angiogenesis was 78.8% and for tumor angiogenesis was 65.19%.

## 1. Introduction

The biological process in which new blood vessels develop from preexisting blood vessels is called angiogenesis [1]. It is a normal process that plays a vital role in the migration, growth, and healing of endothelial cells. Angiogenesis itself is controlled by chemical signals. Usually, the consequences of these chemical signals remain balanced which means that new blood vessels only develop on a need basis. But sometimes these signals can be unbalanced and may increase blood vessel formation, which in return causes abnormal growth or diseases [2, 3]. Angiogenesis plays a vital role in the development and growth of cancer cells [4, 5]. Just like normal cell growth, tumor cells also need oxygen and other nutrients to grow and expand. These elements are present in the blood. Tumor cells send chemical signals that stimulate the growth of new blood vessels. Without the angiogenesis process, abnormal or tumor cells cannot grow beyond 1-2 mm in size [6, 7]. But this abnormal angiogenesis process not only causes cancer but also is a precursor of several diseases like leukemia, hematologic diseases, muscular degeneration, and eye diseases [8–10].

Cancer is ranked as the leading cause of death in the 21st century around the world. According to a survey report published in 2015 by the World Health Organization (WHO), cancer is the first and second major reason for death before the age of 70 in 91 countries around the globe [7]. Furthermore, according to the cancer statistics report 2018 by the International Agency for Research on Cancer and Cancer Research UK, 9.6 million people around the world are dying due to cancer [7, 11]. This ratio is predicted to increase in the coming years.

Researchers, scientists, and biologists all around the world are searching for different techniques for developing different drugs and systems to fight against this deadly disease [12]. Until now, a lot of researchers have contributed their knowledge to develop different systems for tumor prediction at different stages of its life cycle. Different strategies were proposed to control this disease like chemotherapy [13, 14], radiation therapy [15, 16], surgeries, and bone marrow transplant also known as cord blood and vaccines [17]. Cancer can attack the brain that is the most crucial part of the human body. It has the most delicate and complex structure, so it is difficult to inject drugs to cure it. But different approaches can deliver drugs like high-dose chemotherapy, blood-brain barriers, and disruption [18]. Many therapies for tumors revolve around the attempt to suppress the tumor angiogenesis process. Scientists have discovered many ligands that can bind to tumor angiogenesis proteins such that their function is inhibited. Hence, identification of angiogenesis and tumor angiogenesis proteins is crucial in finding novel and effective tumor therapies.

Formerly, several mathematical [3] and computational models have been developed for the classification or identification of various proteomic and genomic attributes [19]. The proposed work establishes a computational model based on position and combinational information of a primary sequence that attempts to accurately identify angiogenesis and tumor angiogenesis proteins. Since tumor angiogenesis proteins are also characterized as angiogenesis proteins, the similarity of their obscure features can often lead to an ambiguous outcome. Ambiguity among seemingly similar angiogenesis and tumor angiogenesis proteins is resolved by a two-layer classification model. The initial layer distinguishes between angiogenesis and nonangiogenesis proteins while the second layer deciphers if a protein identified as an angiogenesis protein is tumor causing or not. The two-layered model helps alleviate ambiguity and yield more accurate and assiduous results.

The rest of the paper is organized as follows.  Section 2 illuminates the importance of angiogenesis uncovered in the previous research and also discusses the state-of-the-art models used for in silico identification of proteomic attributes.  Section 3 discusses the methodology adopted for the proposed in silico identification model.  Section 4 illustrates the accuracy of the model obtained through well-defined rigorous testing methodologies.  Section 5 provides a general discussion regarding the performance of the proposed model.

### 1.1. Current State of the Art

The crucial role of angiogenesis in tumor progression was first discovered by Judah Folkman in 1971 [20]. Angiogenesis is a crucial process of vascular system growth through the sprouting and splitting of blood vessels [21]. Tumor cells also require a constant flow of blood for their growth for which they simulate the growth of blood vessels through secretion of various tumor angiogenesis proteins or growth factors. Cancer treatment therapies are aimed at finding inhibitors for such growth factors. Identification of angiogenesis and tumor angiogenesis proteins bears enormous significance in cancer research as they are targets of such inhibitors [22]. Most of the cancer research revolves around finding ligands and substances that will bind with tumor angiogenesis proteins and inhibit its role [23]. Scientists use various methodologies for the identification of protein attributes [24–28]. In silico identification techniques have evolved and received acclaim over the past few years as they provide robust and fast results and are cost-effective [29, 30]. Scientists have used various mathematical and computational models to identify attributes of proteins based on the composition and positioning of amino acid residues [31]. A position-based mathematical model, namely, position-specific scoring matrix (PSSM), was introduced in 1982 [32]. Numerous prediction models have been designed that incorporate the use of PSSM for the identification of proteomic attributes. However, since PSSM did not incorporate the composition relevant information into the model, therefore it lacked a major aspect that determines proteomic attributes. In 2001, Chou introduced the pseudo amino acid composition model that encompassed position as well as composition information into the model and hence provided better results [33]. Many generalizations and variants have since been proposed to provide even better results [31]. The choice of the most appropriate classifier plays a pivotal role in the design of such methodologies. A multitude of classifiers have been engaged for the prediction of posttranslational modification sites including random forest, support vector machine, neural networks, and deep learning. In [34], the authors incorporate adapted normal distribution biprofile, Bayes, with PseAAC to formulate a prediction model. The accuracy is further improved using kernel sparse representation classification and minimum redundancy and maximum relevance algorithm [35]. Subsequently, an improved depiction uses a deep learning algorithm formulated by [36]. Deep learning has emerged as an encouraging model for the resolution of a multitude of problems [37–39]. The proposed work presents a two-layered model based on position and composition relative features and statistical moments [31] for the identification of angiogenesis and tumor angiogenesis proteins which are probed on various classifiers to accrue the best results.

## 2. Materials and Methods

Angiogenesis has been identified as a critical process that needs to be subjugated to disrupt the progression of cancer. Angiogenesis proteins especially the ones that lead to tumor angiogenesis have a crucial significance in this process. Since they promote the development of new blood vessels within the cancerous tissue, therefore they are considered an important biomarker for early detection of cancer.

Tumors also use the same process for their growth; however, it is possible to uniquely identify the growth factors that are responsible for its growth. In terms of proteomic features, angiogenesis and tumor angiogenesis have mutual properties. Therefore, to fulfill the arduous challenge of distinctly identifying tumor angiogenesis proteins, a two-layered approach is adopted as shown in Figure 1.

The first layer of the model detects whether or not a protein is an angiogenesis protein, using the primary structure of that protein. In the case it is an angiogenesis protein, then the second layer of the model is invoked to decide whether the angiogenesis protein can potentially cause cancer or not.

The proposed workflow is shown in Figure 2, consisting of the following five-step approach; initially, we will collect the well-reviewed and experimentally tested dataset consisting of angiogenesis proteins preprocessed to remove redundancies. Further, feature extractions are performed to transform the biological data into its equivalent mathematical matrix. In the third step, the obtained feature matrix is used to train the model for further prediction. In the fourth step, the model is evaluated for its correctness, sensitivity, specificity, and MCC. In the fifth step, we developed the webserver.

### 2.1. Dataset Collection

The dataset was collected from the UniProt database using meticulously designed search parameters. UniProt is a Universal Protein Resource that contains huge information about the sequence of proteins and their biological functions [22]. A dataset containing positive samples was composed for both angiogenesis and tumor angiogenesis using the UniProt keyword “Angiogenesis.” Similarly, negative samples were also collected. UniProt has no keyword for “Tumor Angiogenesis” proteins. Nonetheless, they comprise within the set of angiogenesis proteins; therefore, tumor angiogenesis proteins were manually curated from the acquired dataset. Each sample within the dataset was manually analyzed for annotated proteomic properties and published evidence within the database to form a set of tumor angiogenesis proteins. However, ambiguous samples were left out. After the collection of data from UniProt, the CD hit suite (http://weizhong-lab.ucsd.edu/cdhit_suite/cgi-bin/index.cgi) was used to reduce the homology of data samples. Clustering of the angiogenesis and tumor angiogenesis datasets was performed by setting the sequence identity parameters at 60%. Ultimately, 761 positive and 2776 negative clusters were formed for the angiogenesis dataset. Similarly, 256 positive and 448 negative clusters were formed for the tumor angiogenesis dataset. A representative sequence was selected from each cluster to form the final dataset.

(1) $$\begin{array}{c} A=A^{+}\cup A^{-}. \end{array}$$

The above equation shows the benchmark dataset used in this work, where *A*^+^ represents the positive data samples of angiogenesis protein and *A*^−^ shows the negative data. Also, the positive tumor angiogenesis samples are represented as *T*^+^, and negative tumor angiogenesis proteins are represented as *T*^−^ as shown in the equation below:

(2) $$\begin{array}{c} T=T^{+}\cup T^{-}. \end{array}$$

### 2.2. Feature Extraction

A robust and efficient methodology for the transformation of biological sequences into a numerical notation for incorporation into a machine learning algorithm is the most pivotal concept in the design of such predictive models [31, 40]. This conversion must keep intact the original information or features of the sequence for analysis in some numerical form. For this purpose, each primary sequence within the collected data is converted into a fixed-size vector. A feature vector of static length is formed which represents a primary sequence and remains essentially invariant upon the scale of the sequence [41]. Incorporation of such a transformation model is ideal as most of the state-of-the-art classifiers work with vectors [22, 42, 43]. A vector described in a model may also lose complete information of the pattern sequence [44]. For this problem, Chou's PseAAC was proposed which is used by many scientists for the construction of genomic and proteomic prediction models and their applications [45, 46]. Later, this model was improved to provide a better correlation perspective among residues that reflect onto feature coefficients.

Let *P* be a sequence of proteins of length *L*, which is represented as

(3) $$\begin{array}{c} P=R_{1}R_{2}R_{3\cdots }R_{16}R_{17}R_{18\cdots }R_{L}, \end{array}$$

where *R*_*i*_ is an arbitrary residue of a polypeptide chain with length *L*.

Feature extraction yields a vector with numerous numerical coefficients. This transformation from a variable-length polypeptide chain into a fixed-length feature vector is illustrated in the following equation:

(4) $$\begin{array}{c} ∆\left(P\right)={\left[\Psi_{1}\Psi_{2}\cdots \Psi_{u}\cdots \Psi_{\Omega }\right]}^{T}, \end{array}$$

where ∆ is the transformation function, Ψ_*i*_ is an arbitrary coefficient, and *Ω* is the constant length of the feature vector [22, 31].

### 2.3. Statistical Moments

The proposed methodology develops on the use of statistical moments to form a numerical representation such that the obscured information within the primary structure of proteins stays intact. These moments form a succinct numerical form such that the original data can be reconstructed without any significant loss of information. Moments can be obtained up to several orders; each provides a deeper perspective into specific aspects of data like positioning, eccentricity, skewness, and peculiarity [31]. Mathematicians and statisticians have devised many moments generating coefficients incarnated based on well-defined distribution functions and polynomials [35, 44].

In the proposed work, Hahn moments, raw moments, and central moments are organized to form a feature set. The Hahn moment bears location- and scale-oriented variance and is calculated based on the Hahn polynomial. Central moments abide information regarding asymmetry, mean, and variance. The central moments are derived for the centroid of collective data making these moments scale variant and location invariant. Subsequently, raw moments are scale and location variants and represent properties like asymmetry, variance, and mean.

A matrix *P*′ with *m* × *m* dimensions is formulated for a two-dimensional residual protein representation where $=\left\lceil \sqrt{L\;}\right\rceil$.

(5) $$\begin{array}{c} P^{\prime }=\left[\begin{array}{ccccc} R_{11} & R_{12} & R_{13} & \cdots & R_{1m}\\ R_{21} & R_{22} & R_{23} & \cdots & R_{2m}\\ \vdots & \vdots & \vdots & \vdots & \vdots \\ R_{m1} & \cdots & \cdots & \cdots & R_{mn} \end{array}\right]. \end{array}$$

The vector *P* is easily transformed into matrix *P*′ by using a simple mapping function explained in [47]. The primary sequence is fitted into a two-dimensional matrix so that it could be formulated into the Hahn polynomial which is orthogonal. The same two-dimensional notation was used for deriving raw and central moments. The Hahn moment is computed using the Hahn polynomial as given below.

(6) $$\begin{array}{c} H_{n}^{v,u}\left(r,N\right)={\left(N+U-1\right)}_{n}{\left(N-1\right)}_{n}\times \overset{n}{\underset{i=0}{\sum }}{\left(-1\right)}^{i}\frac{{\left(-n\right)}_{i}\;\begin{array}{cc} {\left(-r\right)}_{i} & {\left(2N+v+u-n-1\right)}_{i} \end{array}}{\begin{array}{cc} {\left(N+u-1\right)}_{i} & {\left(N-1\right)}_{i} \end{array}}\times \frac{1}{i!}. \end{array}$$

Central moments are computed using the equation given below.

(7) $$\begin{array}{c} \mu_{st}=\overset{k}{\underset{p=1}{\sum }}\overset{k}{\underset{q=1}{\sum }}{\left(p-\bar{x}\right)}^{s}{\left(q-\bar{y}\right)}^{t}P\prime_{pq}. \end{array}$$

The following equation is used to compute the raw moments.

(8) $$\begin{array}{c} M_{st}=\overset{k}{\underset{p=1}{\sum }}\overset{k}{\underset{q=1}{\sum }}p^{s}q^{t}P\prime_{pq}. \end{array}$$

In equations (7) and (8), *s* and *t* represent the order of raw moments. Orthogonality of these moments renders its use assiduous as their inverse functions can be used to reconstruct data. Detailed explanation and use of these notations can be found in [48].

### 2.4. Frequency Vector Determination

The cumulative frequency of occurrence of each specific amino acid residue is furnished into a frequency vector. Information about the distribution of amino acid residues within the primary sequence is summarized into this frequency vector which is represented as

(9) $$\begin{array}{c} FV=f_{1,}\;f_{2,\;}\;f_{3,}\cdots \;f_{20}, \end{array}$$

where **f**_**i**_ refers to the frequency of occurrence of an arbitrary distinct amino acid residue.

### 2.5. Position Relative Incidence Matrix (PRIM) Calculation

The primary sequence of the proteins forms the basis of formulation of feature vectors of primary structures which are otherwise obscure. Information pertaining to position relative incidence of arbitrary protein residues is formulated as a matrix of size (20 × 20). The Position Relative Incidence Matrix (PRIM) is illustrated as

(10) $$\begin{array}{c} X_{PRIM}=\left\lceil \begin{array}{ccc} X_{1,1} & X_{1,2}\cdots & X_{1,j}\cdots \\ \begin{array}{c} X_{2,1}\\ \begin{array}{c} \vdots \\ \begin{array}{c} X_{i,1}\\ \vdots \end{array} \end{array} \end{array} & \begin{array}{c} X_{2,2}\cdots \\ \begin{array}{c} \vdots \\ \begin{array}{c} X_{i,2}\cdots \\ \vdots \end{array} \end{array} \end{array} & \begin{array}{c} X_{2,j}\cdots \\ \begin{array}{c} \vdots \\ \begin{array}{c} X_{i,j}\cdots \\ \vdots \end{array} \end{array} \end{array}\\ X_{N,1} & X_{N,2}\cdots & X_{N,j}\cdots \end{array}\begin{array}{c} \begin{array}{c} X_{1,20}\\ X_{2,20} \end{array}\\ \begin{array}{c} \vdots \\ \begin{array}{c} X_{i,20}\\ \vdots \end{array} \end{array}\\ X_{N,20} \end{array}\right\rceil . \end{array}$$

The sum of the relative position of the *j*th protein residue corresponding to the first occurrence of the *i*th residue is computed in the above matrix given as **X**_**ij**_. The matrix contains all the possible permutations for such occurrences as explained in [48].

### 2.6. Determination of Reverse Position Relative Incidence Matrix (RPRIM)

More obscure features of the primary sequence are uncovered with the help of the Reverse Position Relative Incidence Matrix (RPRIM). The RPRIM is obtained by forming the PRIM of the reversed primary sequence. **X**_**RPRIM**_ is illustrated as

(11) $$\begin{array}{c} X_{RPRIM}=\left\lceil \begin{array}{ccc} R_{1,1} & R_{1,2\cdots } & R_{1,j\cdots }\\ \begin{array}{c} R_{2,1}\\ \begin{array}{c} \vdots \\ \begin{array}{c} R_{i,1}\\ \vdots \end{array} \end{array} \end{array} & \begin{array}{c} R_{2,2\cdots }\\ \begin{array}{c} \vdots \\ \begin{array}{c} R_{i,2\cdots }\\ \vdots \end{array} \end{array} \end{array} & \begin{array}{c} R_{2,j\cdots }\\ \begin{array}{c} \vdots \\ \begin{array}{c} R_{i,j\cdots }\\ \vdots \end{array} \end{array} \end{array}\\ R_{N,1} & R_{N,2\cdots } & {\text{R}}_{N,j\cdots } \end{array}\begin{array}{c} \begin{array}{c} R_{1,20}\\ R_{2,20} \end{array}\\ \begin{array}{c} \vdots \\ \begin{array}{c} R_{i,20}\\ \vdots \end{array} \end{array}\\ R_{N,20} \end{array}\right\rceil , \end{array}$$

where **R**_**i**,**j**_ is an arbitrary element of **X**_**RPRIM**_.

### 2.7. Accumulative Absolute Position Incidence Vector (AAPIV) Calculation

The AAPIV matrix is used to calculate the sum all the positions at which each native amino acid occurs within the primary sequence; hence, it bears a length of 20 and is denoted as

(12) $$\begin{array}{c} AAPIV=\left[v_{1},v_{2\;},v_{3},\cdots v_{20}\right]. \end{array}$$

Any *i*^th^ element in the above matrix is computed as

(13) $$\begin{array}{c} v_{i}=\overset{n}{\underset{k=1}{\sum }}P_{k}, \end{array}$$

where *P*_*k*_ is the position of occurrence of a native amino acid while *n* is its frequency of occurrence.

All the above-defined features are aggregated to form a feature vector. The dimensionality of *P*′, *X*_PRIM_, and *X*_RPRIM_ is reduced by computing their Hahn, central, and raw moments. Ultimately, a fixed-size feature vector is formed to represent primary structures of varied lengths.

## 3. Prediction Algorithm

After extraction of feature vectors from positive as well as negative sequences, the data is used to train classifiers. A diverse set of currently widespread classifiers were used for the purpose which includes random forest, neural network, and support vector machine. Comparison of results yielded from each classifier work enables the identification of the most suitable classifier with the highest accuracy.

### 3.1. Random Forest

The random forest (RF) classifier was trained at two levels for the prediction of angiogenesis and tumor angiogenesis proteins. At the first level, the classifier was used to identify angiogenesis and nonangiogenesis proteins while at the second level the angiogenesis protein was passed through another classifier to identify if the protein is tumor causing or not. The random forest is a very powerful classifier used for classification and regression problems [49, 50]. Initially, it converts the whole data into decision trees [23, 51]. Furthermore, a random forest classifier is applied to each tree to predict a class. The class with the highest votes becomes the models' prediction result [41] as illustrated in Figure 3.

### 3.2. Artificial Neural Network (ANN)

Subsequently, the artificial neural network (ANN) was also similarly employed at two levels. ANN has interconnected layers of neurons [52]. The connectionist architecture of the backpropagation network is illustrated in Figure 4. The ANN mechanism used is based on a feedforward network and uses the backpropagation algorithm to reduce error. An input layer is clamped to the input feature vectors. It also has a hidden layer that receives selected numbers of neurons from the input layer and forms the main processing unit of the whole network. The activation unit of ANN sums all preceding weighted inputs in addition to bias values [23, 31]. The output of the 3-layer feedforward network with error backpropagation is represented by

(14) $$\begin{array}{c} O_{m}=f\left(\overset{h}{\underset{y=1}{\sum }}W_{ym}\times f\left(\overset{k}{\underset{x=1}{\sum }}W_{xy}I_{a}\right)\right), \end{array}$$

where the input layer has *k* neurons and the hidden layer has *h* neurons. Partial output calculated by the *m*th neuron in the network is denoted by *O*_*m*_. Supposing that the arbitrary node receives an input *I*_*a*_, then *W*_*xy*_ represents the weight of the edge connecting node *x* to node *y*. Similarly, *W*_*ym*_ represents the weight of the *y*th node connected to an arbitrary output layer neuron *m*. The classical sigma function which determines the activation of neurons is denoted as *f* in

(15) $$\begin{array}{c} f\left(x\right)=\frac{1}{\left(1+e^{-x}\right)}. \end{array}$$

Actual activated levels in the output units are compared with the target output for every training iteration. The error rate hence observed is denoted by ∈ and is calculated by the difference between the expected output and actual activated output given as

(16) $$\begin{array}{c} \in =0.5\overset{o}{\underset{i=1}{\sum }}\left(O_{i}-P_{i}\right), \end{array}$$

where *O*_*i*_ is the target output, *P*_*i*_ is the actual calculated output by the network, and *o* is the number of neurons in the output layer. The gradient descent method is used to minimize the error rate. The error generated at the output layer is sent back to the input layer. The set of all the weights is represented by a vector *V*. The backpropagation procedure selects a differential ∆*V* such that it lessens the error. This is continued iteratively until convergence is achieved as shown below:

(17) $$\begin{array}{c} V\left(t+1\right)=V\left(t\right)+∆V\left(t\right), \end{array}$$

where

(18) $$\begin{array}{c} ∆V=\eta \left(-\frac{\partial \in }{\partial W}\right)\left|V=V\left(t\right)\right.. \end{array}$$

This equation shows a change in weight at time *t* + 1, and a positive constant *η* signifies the learning rate usually set between 0 and 1. The change in weights is expressed as

(19) $$\begin{array}{c} \Delta V_{u,v}=-\eta \frac{\partial \in }{{\partial W}_{u,v}}. \end{array}$$

Here, Δ*V*_*u*,*v*_ shows the minimal ∈ weight among the *u*^th^ and *v*^th^ neurons in the *i*^th^ iteration. This procedure is followed in both backward and forward passes of input signals. It is a lightweight procedure that consumes less memory space, and it is extensively used for the training of ANN. Patterns are repetitively offered to the network to train it and to make it capable of minimizing the mean square error (MSE) as shown in

(20) $$\begin{array}{c} \text{MSE}=\frac{1}{2n}\overset{n}{\underset{j=1}{\sum }}\overset{k}{\underset{i=1}{\sum }}{\left(P_{i}^{o}-O_{i}^{o}\right)}^{2}. \end{array}$$

The actual output received at the *i*^th^ neuron of the output layer is represented as *O*_*i*_^*o*^, and *P*_*i*_^*o*^ represents the expected value where the total number of input samples is *n* and there are *k* output neurons.

### 3.3. Support Vector Machine (SVM)

A support vector machine (SVM) is a machine learning classifier that is used in regression-related problems. SVM works by attempting to fit in a hyperplane in an *N*-dimensional space where *N* represents the number of feature elements that represents the samples distinctly. Hyperplanes are simple decision boundaries that classify the data points, and these data points are present on both sides of the hyperplane, which ideally partitions different classes. The hyperplane is most optimally adjusted by means of support vectors.  Figure 5 illustrates points on either side of the hyperplane belonging to different classes, namely, class A and class B.

## 4. Results and Discussion

### 4.1. Evaluation of the Model

In the current study, the dataset was constructed on two levels. The first level uses 785 positive and 2776 negative samples regarding angiogenesis proteins whereas the second level encompasses 256 positive and 448 negative samples for tumor angiogenesis proteins. A feature vector input matrix (FIM) was formed for both angiogenesis and tumor angiogenesis datasets separately. Every single row of FIM is a feature vector that represents a single data sample. Also, an Expected Output Matrix (EOM) was formed corresponding to FIM. All the classifiers were trained using both FIM and EOM. FIM was given as an input for training the model where EOM was used to compute errors and retrain until convergence is achieved [23, 31, 43, 45].

All the classifiers were implemented using Python version 3.6 using SciKit Learn API. Subsequently, results gathered using this framework are rigorously analyzed in terms of their performance parameters.

A major design issue regarding the design of a new prediction model is to set up some parameters to measure its accuracy. Researchers have predominantly used four descriptive metrics for performance analysis. These metrics are as follows:

1. Sp measures the specificity which quantifies the ability of the model to identify positive samples accurately [46]
2. Sn measures the sensitivity, which represents the accuracy in predicting negative data samples
3. Acc is used to measure the overall accuracy of the model
4. MCC is for measuring the stability of the model
5. The following formulation is used to quantify these metrics.

(21) $$\begin{array}{c} \text{Specificity }\left(\text{Sp}\right)=\frac{\text{TN}}{\left(\text{TN}+\text{FP}\right)}, \end{array}$$

(22) $$\begin{array}{c} \text{Senstivity }\left(\text{Sn}\right)=\frac{\text{TN}}{\left(\text{TP}+\text{FN}\right)}, \end{array}$$

(23) $$\begin{array}{c} \text{Accuracy}\left(\text{Acc}\right)=\frac{\left(\text{TP}+\text{TN}\right)}{\left(\text{TP}+\text{FP}+\text{TN}+\text{FN}\right)}\times 100, \end{array}$$

(24) $$\begin{array}{c} \text{MCC}=\frac{\left(\text{TP}\right)\left(\text{TN}\right)-\left(\text{FP}\right)\left(\text{FN}\right)}{\sqrt{\left(\text{TP}+\text{FN}\right)\left(\text{TN}+\text{FP}\right)\left(\text{TP}+\text{FP}\right)\left(\text{TN}+\text{FN}\right)}}, \end{array}$$

where true negatives are represented by TN, true positives are represented by TP, false positives are represented by FP, and false negatives are represented by FN [43, 53, 54].

But unfortunately, the formation of equations (21), (22), (23), and (24) is somewhat cryptic for biologists [55]. Another more intuitive format has been suggested by scientists in [56, 57], and their modifiers were introduced in [47]. Symbols used to represent these equations are *N*^+^, *N*^−^, *N*_−_^+^, and *N*_+_^−^. Explanation of these representations is given in Table 1.

Hence, these metrics are also calculated as

(25) $$\begin{array}{c} \left\{\begin{array}{c} \text{Sn}=1-\frac{N_{+}^{-}}{N^{+}},\\ \text{Sp}=1-\frac{N_{+}^{-}}{N^{-}},\\ \text{Accuracy}=1-\frac{N_{-}^{+}+N_{+}^{-}}{N^{+}+N^{-}},\\ \text{MCC}=\frac{1-\left(\left(N_{-}^{+}/N^{+}\right)+\left(N_{+}^{-}/N^{-}\right)\right)}{\sqrt{\left(1+\left(\left(N_{+}^{-}-N_{+}^{-}\right)/N^{+}\right)\right)\left(1+\left(\left(N_{-}^{+}-N_{+}^{-}\right)/N^{-}\right)\right)}}. \end{array}\right. \end{array}$$

### 4.2. Validation Methods

Testing is another important factor for the validation of the predicting models [22, 31, 42, 45]. The validation phase encompasses four most commonly used tests discussed below.

#### 4.2.1. Self-Consistency

The self-consistency test is the most trivial and intuitive of the tests. A trained model is simply tested on the dataset that was used to train it. Capability of a model to learn from a given dataset is underscored with this basic but useful evaluating benchmark. Good results merely indicate that the classifier has the ability to find obscure patterns within the training data. Self-consistency testing was performed on angiogenesis and tumor angiogenesis datasets upon which the proposed model was trained. Results obtained from self-consistency tests are illustrated in Table 2 showing the overall performance of the proposed model using random forest (RF), artificial neural network (ANN), and support vector machine (SVM) classifier.

The results indicate that the random forest classifier has the best capability to learn and decipher obscure patterns that peculiarly characterize each sample.

#### 4.2.2. Cross-Validation

The cross-validation technique is used when unknown data for testing is not readily available [45, 58]. The dataset is randomly divided into multiple partitions or folds spanning over a comprehensive sample space hence rendering cross-validation as a rigorous test. Partitions are devised in a manner such that they are disjointed from each other and are comparable in size. A partition is left out while the model is trained on the rest of the data. Once the model is fully trained, the left-out partition is used as unknown data to test the model. These steps are recapitulated for each fold. The overall accuracy of the model for the cross-validation test is reported by taking the mean of accuracy yielded against each fold.

Cross-validation tests were performed by partitioning the benchmark dataset into 5-folds and 10-folds.  Table 3 depicts the results of the test.

The random forest exhibits the best results at both levels with an accuracy of 99.7% for the identification of angiogenesis proteins and an accuracy of 99.5% for the identification of tumor angiogenesis proteins.

#### 4.2.3. Jackknife Testing

Jackknife testing is the most rigorous testing methodology. In each iteration, it leaves out a single sample while the model is trained on the rest. After sufficient training, the model is tested with the left-out sample. This process exhaustively proceeds for all data samples. Hence, this test is repeated *N* times, where *N* represents the size of the overall dataset. In every iteration, the testing data sample is different, so all samples are tested exactly once. This technique is the most rigorous which also makes it slower [59–63]. After successfully training and testing, the number of true positive, false positive, true negative, and false negative was obtained [55].

Since the sample is tested exactly once, therefore the overall accuracy obtained for this test remains unique [31, 40, 45, 46].

RF results illustrated in Table 4 for angiogenesis and tumor angiogenesis proteins portray higher accuracies and are reported as 99.3% and 99.7%, respectively, in comparison with other classifiers.

#### 4.2.4. Independent Set Testing

Independent test evaluates how well a model performs on unknown data. Initially, the data is partitioned such that the larger partition is used for training and the left-out partition is used as unknown data for testing. Once the model is completely trained, then independent set testing is performed using the left-out data. An independent set needs to be formulated intelligibly such that the training data encompasses comprehensive obscure patterns and the test data thoroughly queries the ability of the model to decipher these patterns. Otherwise, testing results may be ambiguous. Results obtained from independent testing illustrate the overall accuracies of RF, ANN, and SVM classifiers after independent testing as presented in Table 5.

The random forest shows the best results as compared to ANN and SVM classifiers at both levels for the identification of angiogenesis as well as tumor angiogenesis proteins while the performance of the ANN classifier is better than that of the SVM classifier.

Working with classification models renders performance measurement as an essential task quantified using classification scores. But this type of performance is not suitable while dealing with flawed datasets with heavy class imbalance. In such cases, ROC (Receiver Operating Characteristic) curves provide a graphical view along with quantitative analysis of the overall scenario. ROC is a prevalently used performance evaluation method for evaluating any classification model. The ROC curve is plotted by mapping the True Positive Rate (TPR) against the False Positive Rate (FPR). It depicts the accuracy with which the model is capable of distinguishing among classes. TPR is plotted along the *y*-axis while FPR is plotted along the *x*-axis. Estimation of the area under the curve is a measure of the model's performance. The best possible accuracy is 1, and the worst is 0.5. A good measure of separability means that the model has accuracy near 1, and similarly, accuracy near 0 indicates that the model has the worst measures of separability. Consequently, an accuracy of less than 0.5 indicates that the model will perform exactly the opposite of what a model was recommended to do.

Various testing techniques were applied to gauge the effectiveness of the classifiers as discussed earlier. To prioritize the classifiers based on efficiency, a comparison is depicted through a ROC curve.  Figure 6 represents the comparison based on testing performed in the previous section. Figures 6–10 depict that RF shows the best results in comparison with ANN and SVM. The RF curve encompasses an area close to 1 implying that the model has the best measure of separability. Graphical representations accentuate that RF and ANN both exhibit better results as compared to SVM. However, in the case of jackknife testing, SVM classifier accuracy is high as compared to that of ANN as illustrated in Figure 10.

A similar comparison is performed for classifiers at the second level which predicts tumor angiogenesis proteins. Figures 11–15 illustrate the results of various test techniques performed on the tumor angiogenesis dataset. These figures connote that the RF classifier exhibits better results in comparison with the ANN and SVM classifier supported by the fact that the area under the RF curve is approximately approaching 1.

## 5. Webserver

Formulation of the robust dataset and feature extraction methodology forms the foundation of a computationally intelligent model for efficient prediction of uncategorized proteomic sequences. However, the availability of such a tool is also of extreme importance so that the research community could benefit from it [45]. To make a novel predictor for the forbearance of all users and biologists around the globe, there is a need for a user-friendly and publically accessible webserver. In the final step of Chou's 5-step rule, a webserver is devised for this purpose [48]. The webserver enables scientists and biologists to easily access and to utilize such prediction applications without getting into the complex mathematical details. The webserver for the proposed work will soon be made available. Meanwhile, its code has been made available along with a readme file at https://github.com/RabiaKhan-94/Thesis_WebServer.git which can be easily set up by an intermediate-level Python developer.

## 6. Discussion and Conclusion

This study proposes a prediction model for the classification of angiogenesis and tumor angiogenesis. A robust well-defined methodology was adopted for dataset collection. Duplicate and redundant data were removed, and homologous sequences up to 60% were excluded. Variable-length proteomic sequences were transformed into fixed-length feature vectors using a position- and composition-based technique. Position relative information was further transmuted into a succinct form using statistical moments. Three classifiers random forest (RF), artificial neural network (ANN), and support vector machine (SVM) were used to find the best results. All of these algorithms are powerful, robust, and well understood. The random forest (RF) and artificial neural network (ANN) can deal with linear as well as complicated nonlinear problems. The current study reveals that RF showed the best results among these classification approaches. As a result of cross-validation, RF exhibited an accuracy of 97.8% for angiogenesis proteins and an accuracy of 99.5% for tumor angiogenesis, where ANN showed an accuracy of 99.1% for angiogenesis and 79.9% for tumor angiogenesis. Additionally, the accuracy of SVM for angiogenesis was 78.8%, and for tumor angiogenesis, it was 65.19%. The current study has shown different performances for all approaches. Consequently, it concludes that the results exhibited by RF are better than ANN and SVM. On the other hand, the random forest takes less time for training as compared to the neural network. Another important strength of RF is that it is less susceptible to overfitting which is not the case with a neural network. The robustness of the feature extraction technique plays a significant role in the overall accuracy of the model. Feature extraction uncovers obscure features more pertinent to the composition and sequence of the primary structures. The meticulously collected data helps the model to produce better results. The in silico nature of the model makes it an alluring opportunity as it is timely and cost-effective. Biologists and scientists can greatly benefit from the proposed tool for the characterization of proteins and understand their role in angiogenesis and tumor angiogenesis processes. Furthermore, the model can prove to be effective in identifying the biomarkers that cause a tumor. Additionally, it augments the work of biologists and scientists in research aimed at finding new treatments and discovering new drugs.

Tumor-causing angiogenesis proteins are important biomarkers for the onset of cancer. Timely identification of these proteins can help in the treatment and possible cure of the disease. This study proposes a robust in silico technique for the identification of tumor angiogenesis using a two-level predictor. The first level indicates whether a protein is an angiogenesis protein or not while the second level identifies whether the given protein is responsible for tumor angiogenesis or not. A mature feature extraction technique was used to gather features for the benchmark dataset. Classifiers like RF, SVM, and ANN were trained using the resultant feature vectors. Once the models are thoroughly trained, they are rigorously tested using test methods like *k*-fold cross-validation, self-consistency, independent set testing, and jackknife testing. The random forest classifier showed 99.3% accuracy for angiogenesis and 99.7% for tumor angiogenesis, and ANN showed an overall 96.23% accuracy for angiogenesis and 95% for tumor angiogenesis. On the other hand, SVM showed 78.65% accuracy for angiogenesis and 65.19% for tumor angiogenesis.

## 7. Future Works

Advanced drug therapies and treatments integrate the use of ligands that target tumor angiogenesis proteins to inhibit them. Inhibition of these tumor growth factors disrupts its growth, and in some cases, the tumor even dies out. Tools that help the discovery and identification of tumor angiogenesis proteins greatly help cancer researchers to identify these growth factors in a timely and cost-effective manner. One such tumor growth factor has been uncovered; there is an incessant need to identify ligands that can inhibit them. In silico models that simulate ligand bindings with tumor growth factors can also greatly enhance tumor research. Further, in the future, the proposed model can be made more adaptive by incorporating updated data and using deep learning features.

## Figures and Tables

**Figure 1:** Flowchart of the proposed system.

**Figure 2:** The workflow of the proposed model is shown which includes five steps: data collection and its preprocessing, feature extraction, training, model evaluation, and the construction of the webserver.

**Figure 3:** Random forest classifier architecture.

**Figure 4:** Architecture of ANN.

**Figure 5:** Architectural diagram of SVM.

**Figure 6:** Comparison based on self-consistency.

**Figure 7:** Comparison through 5-folds.

**Figure 8:** Comparison based on 10-folds.

**Figure 9:** Jackknife testing comparison.

**Figure 10:** Independent testing comparison.

**Figure 11:** Comparison based on self-consistency.

**Figure 12:** Comparison based on 5-folds.

**Figure 13:** Comparison based on 10-folds.

**Figure 14:** Comparison of jackknife testing.

**Figure 15:** Comparison based on independent testing.

**Table 1:** New symbol description for Chou's fourth step.

Symbols	Explanation
*N* ^+^	Represents the total number of true positives in the dataset
*N*_−_^+^	The total number of true positives in the dataset projected incorrectly
*N* ^−^	The total numbers of true negatives in the dataset
*N*_+_^−^	The total number of negatives projected incorrectly

**Table 2:** Self-consistency results for angiogenesis and tumor angiogenesis.

	Angiogenesis								Tumor angiogenesis							
Predictor	TP	FP	TN	FN	Acc (%)	Sp (%)	Sn (%)	MCC	TP	FP	TN	FN	Acc (%)	Sp (%)	Sn (%)	MCC
RF	783	0	2784	0	100	100	100	1	255	1	447	1	99.7	99.6	99.8	0.9
ANN	766	7	2580	204	94.1	99.1	92.7	0.9	256	0	307	141	79.9	100	68.5	0.6
SVM	31	752	2783	1	78.9	4	100	0.2	12	244	447	1	65.2	4.7	99.8	0.2

**Table 3:** *k*-fold cross-validation results.

	Level 1									Level 2							
Predictor	Fold	TP	FP	TN	FN	Acc (%)	Sn (%)	Sp (%)	MCC	TP	FP	TN	FN	Acc (%)	Sn (%)	Sp (%)	MCC
RF	**5**	723	60	2784	0	98.1	92.3	100	0.95	254	2	448	0	99.7	99.2	100	0.9
ANN		653	130	2780	4	96.2	83.4	99.9	0.8	246	10	428	20	95.7	96.1	95.7	0.9
SVM		31	752	2783	1	78.8	4	100	0.2	6	250	448	0	64.5	2.3	100	0.1
RF	**10**	706	77	2784	0	97.8	99.4	100	0.9	253	3	0	448	99.5	98.8	100	0.9
ANN		776	7	2580	240	94.1	99.1	92.7	0.8	256	0	307	141	79.9	100	68.5	0.7
SVM		31	752	2783	1	78.8	4	100	0.2	12	244	447	1	65.19	4.7	99.8	0.2

**Table 4:** Jackknife results.

	Angiogenesis								Tumor angiogenesis							
Model	TP	FP	TN	FN	Acc (%)	Sn (%)	Sp (%)	MCC	TP	FP	TN	FN	Acc (%)	Sp (%)	Sn (%)	MCC
RF	781	26	2784	0	99.3	100	100	1	255	1	447	1	99.7	99.6	99.8	0.9
ANN	653	130	2780	4	96.3	83.3	99.9	0.8	246	10	428	20	95.7	96.1	95.5	0.9
SVM	783	0	2784	0	100	100	100	1	6	250	448	0	64.5	2.3	100	0.1

**Table 5:** Independent set results.

	Angiogenesis								Tumor angiogenesis							
Model	TP	FP	TN	FN	Acc (%)	Sn (%)	Sp (%)	MCC	TP	FP	TN	FN	Acc (%)	Sp (%)	Sn (%)	MCC
RF	211	27	833	0	94.5	88.7	100	0.9	70	0	142	0	100	100	100	1
ANN	227	14	827	3	98.4	94.2	99.6	0.9	59	12	141	0	94.3	83.1	100	0.9
SVM	3	238	833	7	77.2	1.2	99.2	0.02	5	66	131	10	64.2	7.0	92.9	0.01

## Data Availability

Data is available at https://github.com/RabiaKhan-94/Angio_Webserver.
